# Machine Learning Algorithms for Prediction of Survival Curves in Breast Cancer Patients

**DOI:** 10.1155/2021/9338091

**Published:** 2021-11-20

**Authors:** Roqia Saleem Awad Maabreh, Malik Bader Alazzam, Ahmed S. AlGhamdi

**Affiliations:** ^1^Prince Al Hussein Bin Abdulla, Academy for Civil Protection, Jordan; ^2^Faculty of Computer Science and Informatics, Amman Arab University, Jordan; ^3^Department of Computer Engineering, College of Computers and Information Technology, Taif University, P.O. Box 11099, Taif 21944, Saudi Arabia

## Abstract

Today, cancer is the second leading cause of death worldwide, and the number of people diagnosed with the disease is expected to rise. Breast cancer is the most commonly diagnosed cancer in women, and it has one of the highest survival rates when treated properly. Because the effectiveness and, as a result, survival of the patient are dependent on each case, it is critical to know the modelling of their survival ahead of time. Artificial intelligence is a rapidly expanding field, and its clinical applications are following suit (having surpassed humans in many evidence-based medical tasks). From the inception of since first stable risk estimator based on statistical methods appeared in survival analysis, there have been numerous versions of it created, with machine learning being used in only a few of them. Nonlinear relationships between variables and the impact they have on the variable to be predicted are very easy to evaluate using statistical methods. However, because they are just mathematical equations, they have flaws that limit the quality of their output. The main goal of this study is to find the best machine learning algorithms for predicting the individualised survival of breast cancer patients, as well as the most appropriate treatment, and to propose new numerical variable stratifications. They will still be carried out using unsupervised machine learning methods that divide patients into groups based on their risk in each dataset. We will compare it to standard groupings to see if it has more significance. Knowing that the greatest challenge in dealing with clinical data is its quantity and quality, we have gone to great lengths to ensure their quality before replicating them. We used the Cox statistical method in conjunction with other statistical methods and tests to find the best possible dataset with which to train our model, despite its ease of multivariate analysis.

## 1. Introduction

Cancer is the second leading cause of death worldwide, with an estimated 9.6 million deaths in 2018 (1 in 6 deaths), and the cases of diagnosis and deaths from it continue to increase each year [1]. Survival analysis is very popular due to its simplicity, and, in addition to being used in medical statistics, it has extensive application in other fields such as economics, education, biology, or industry. The nonpayment of a credit when an electrical appliance stops working and the abandonment of studies by a student are some of the events that are studied with this technique. Its main application in medicine is to analyze events of interest: death, relapse, adverse reaction to a drug, or the development of a new disease. For all these cases, it is possible to model and know the risk of the event taking place in a range of time from weeks to years depending on the case. There are many predictors that have been developed to estimate the individual risk of women with breast cancer. Some of the best known and accepted in a standard way are the Gail model by Gail MH in 1989 [2]. The survival analysis aims to model the time that elapses until a certain event occurs, relating the outcome of a patient with its associated descriptive biological variables. In recurrence prediction studies, although, as in the previous case, statistical methods prevail [3, 4]. With some difficulty, we can find some studies that have applied computational learning [5], and the precision results of these increase significantly. In this project, we will analyze the behaviour of automatic learning models to predict death and recurrence against statistical methods, while we will take advantage of the advantages that the latter offer to select a set of variables. Optimal with which to train our model, a task in which they have given very good results over time.

## 2. Material and Methods

In the development of this project, we have worked in parallel with two sets of survival data Hospital and Attributes.

1. Hospital dataset of patients with hormone receptor-positive breast cancer treated with adjuvant hormonal therapy, free of disease 5 years after the first diagnosis. They were taken from the Baghdad Teaching Hospital (Iraq). From these, we will analyze their probability of recurrence
2. Patient samples

*Numerical variables*. Age 67 years on average, number of lymph nodes affected, number of lymph nodes removed, tumor size (in mm), and follow-up time (in years).

*Categorical variables*. Menopausal status (premenopausal, postmenopausal), grade (I, II, and III), hormonal receptors (estrogen, progesterone, and her2), cancer subtype (Luminal A and Luminal B), risk (low, medium, and high), hormonal therapy (aromatase inhibitors (AI), Tamoxifen, and AI+Tamoxifen), last control state (dead with disease, dead without disease, alive with disease, and alive without disease), hormone receptor (created from hormone receptors: positive in estrogen and progesterone, positive in estrogen), and event (in this case, it means recurrence, with values 0 and 1).

*TCGA*. We obtained this dataset, also from breast cancer patients, from The Cancer Genome Atlas [6], a public library with data on 33 types of cancer. For this, we have made use of the TCGA retriever library in R [7]. From these, we will analyze their probability of death.

*Software*. All the software implemented in this project has been made in R, using RStudio. The packages used mainly have been mentioned throughout the methodology (survival, tcga, mlr, h2o, ...). The developed software is uploaded in the public repository https://github.com/nairachiclana/ML_and_Survival-BreastCancer in the form of .rmd files except for the code corresponding to the interface. The data from the TCGA set is extracted in the code; the data from the Hospital set cannot be shared due to data protection.

*Hardware*. I have used my personal machine, macOS Mojave software version 10.14.5 with 8GB RAM, 1 TB of hard disk, and an Intel Core i5 3.4 GHz processor. Since the high-compute algorithms have been trained using the parallelization offered by h2o as mentioned above, the team has not assumed any limitations.

### 2.1. Methods

The objective is to find predictors of survival for each dataset and to be able to visualize the curves predicted from input variables in an interface. The first step is to prepare the data; for this, using statistical methods, we will evaluate which stratification is more adequate. It is the next step to cleaning data and essential for the proper functioning of machine learning algorithms. We will apply correlation analysis and confirm this by hypothesis tests in case it is necessary to eliminate any of this final set.

### 2.2. Variable Creation

The groupings that we will build and evaluate, in addition to those defined by the clustering algorithms, will be, in the variables that allow it, those defined by the paper that we replicate as the first task of this project [8] and those commonly used in medical practice. We can see them in Table 1.

We know that the proper functioning of a clustering algorithm depends largely on the spatial distribution of the data. In the Hospital dataset and TCGA dataset, we can see that the distribution of the variables to cluster is within normality and we do not have to use any specific algorithm that adapts to themselves. For these distributions, we will use the general-purpose algorithms K-means and hierarchical, evaluating them previously to see which one is best suited in each case.

To decide the number of clusters and algorithm used in each variable, we will follow the following procedure:

1. View the silhouette index and elbow method values for each *k* ∈ (1, 10]
2. See, for each value of *k* (in a set more reduced to the previous one) and algorithm, the values of silhouette index, Dunn index, and connectivity. Here, we will see, according to each index, the number of clusters and the most suitable method for the variable in question
3. In case the choice is hierarchical, we evaluate the silhouette index for the different measure average, complete and single
4. Once the number of clusters and algorithm have been decided, we make the partitions, check that there are no excessively unbalanced levels, and visualize them in the distribution histogram

### 2.3. Cluster Hospital

- Age: K-means with *k* = 4; (0.44], (44.56], (56.69], and (69,100] contain 134, 249, 266, and 178 records, respectively
- Lymph nodes affected: K-means with *k* = 2; [0,4] and (4,25] contain 743 and 84 records, respectively. Hierarchical with 2 clusters in addition to separating the value 0 and single measure; 0, (0,10], and (10,25] contain 415, 349, and 27 records, respectively
- Lymph nodes extracted: hierarchical with 4 clusters and average size; [0,1], (1,11], (11,17], and (17,32] contain 183, 290, 222, and 131 records, respectively
- Tumor size: hierarchical with 2 clusters and average size; (0,27] and (27,60] contain 672 and 155 records, respectively. K-means with *k* = 3; (0,12], (12,31], and (31,58] contain 373, 328, and 126 records, respectively
- Ki67: hierarchical with 7 clusters and average measure; (0.11], (11.20], (20.31], (31.40], (40.49], (49.56], and (56.63]) contain 262, 182, 131, 76, 100, 39, and 37 records, respectively

TCGA clusters

- Age: K-means with *k* = 4; (0.45], (45.57], (57.70], and (70.100] contain 105.202, 211, and 130 records, respectively. K-means with *k* = 3; (0.54], (54.70], and (70,100] contain 263, 255, and 130 records, respectively
- Lymph nodes affected: K-means with *k* = 4; [0,5], (5,12], (12,21], and (21,44] contain 319, 126, 130, and 73 records, respectively. K-means with *k* = 3 in addition to the value 0; 0, (0,8], (8,19], and (19,44] contain 95, 273, 196, and 84 records, respectively

For the variable that indicates the number of affected lymph nodes, due to the high concentration of the value 0 in both sets (55% of the data in Hospital and 15% in TCGA), we have created a single set with this value in addition to those indicated by the algorithm.

### 2.4. Analysis and Choice of Variables

Following the 3 different distributions of numerical variables, we have defined from each initial dataset (Hospital and TCGA) and having in common the categorical variables, 3 different datasets:

*Standard*: contains the numerical variables corresponding to the standard grouping (defined in Table 1). Only for the Hospital complex.

*Combined*: for each numerical variable, we will choose a stratification between standard, paper, and defined by cluster algorithms based on the *p* value and 95% CI given by Kaplan-Meier and Cox PH.

Once the different datasets referring to the two original datasets are formed, we will evaluate whether they fulfill the Cox proportional hazards test and the Cox test of global significance of variables, thus being able to choose the combination of more variables suitable for each outfit. All the statistical measures and tests were mentioned. The statistical methods (Cox PH and Kaplan-Meier).

### 2.5. Hospital Set

#### 2.5.1. Statistical Analysis of Stratifications

For all cases, although the ones with the lowest *p* value according to both estimators are disaggregated, their confidence intervals are very wide, so we will discard them as quality options. In the following, we see the stratifications of each variable ordered from highest to lowest quality contributed to the set, the first being the one chosen to form part of the combined dataset. For this classification, we are based on the values in Table 2.

- Age: K-means *k* = 4, standard
- Lymph nodes affected: hierarchical *k* = 3, paper and standard, K-means *k* = 2
- Lymph nodes extracted: hierarchical *k* = 4
- Tumor size: paper, K-means *k* = 3, standard, hierarchical *k* = 2
- Ki67: paper, standard, hierarchical *k* = 7

#### 2.5.2. Cox Proportional Hazards Test

One of the assumptions made by this model is the proportionality of risks. We will check if our sets comply with it, having to discard them otherwise. We are based from the beginning on the null hypothesis that proportionality is fulfilled. In case the global *p* value is less than 0.05, we will have to discard this hypothesis and accept that it is not fulfilled.

In Table 3, we can see that proportionality is fulfilled for the three sets. We can also see that according to the Chi estimator, none reject the independence hypothesis, although the one most likely to do so would be paper.

#### 2.5.3. Cox Global Significance Test

The results are the same for the LogRank and likelihood tests. We found a slight difference in the Wald test in favor of the combined set, indicating that this set of variables is more significant. We can see it in Tables 3 and 4.

For this reason, the combination of variables chosen to represent the Hospital set is combined.

### 2.6. TCGA Set

#### 2.6.1. Statistical Analysis of Stratifications

Age: K-means *k* = 3, K-means *k* = 4, standard.

Lymph nodes affected: K-means *k* = 3, standard, K-means *k* = 4.

We see the details of this classification in Table 5.

#### 2.6.2. Cox PH Proportional Hazards Test

After doing the test the first time, we had to eliminate the variable stage because it did not fulfill the independence of time. In addition, it had a very low *p* value that unbalanced the mean making the global one have a value of 1. Once this variable has been eliminated, although the *p* value is the same for the two sets, the Chi estimator tells us that in standard rejects the null hypothesis of independence of variables. Combined, however, it does have a set of variables that provide different information (Table 6).

#### 2.6.3. Cox PH Global Significance Test

In the Wald test (against a coincidence of values in LogRank and likelihood), we confirm that combined has more global significance than standard (Table 6).

For this reason, the combination of variables chosen to represent the TCGA set is combined.

*Correlation and hypothesis.* Using the Spearman 2.1.4 correlation coefficient, we will see the association strength of the variables to check if it is convenient to eliminate some that are highly correlated with another from the final set. We will study the hypotheses of the possible correlations observed by the Spearman index. Hypothesis tests are performed using the survdiff function [9] that evaluates the difference between survival curves. We understand *H*_0_ as the independence of variables.

*Hospital complex*. We see the correlations and the corresponding result of the hypothesis test in Table 7. The independence test is not fulfilled for tumor size and risk, yet we decided not to eliminate them because the correlation index is not too high (0.51) and both have some correlation with the event variable as shown in Table 8. We did not observe any significant inverse correlation.

TCGA set. We see the correlations and the corresponding result of the hypothesis test in Table 9. By the hypothesis test, we accept the correlation between menopause and age, but as before, at not be a correlation with too high an index, and in this case having a very small total number of variables, we will not eliminate any of them.

Final sets Hospital set: Tables 10 and 11.

The median survival rate is zero because survival never reaches the value 0.5 (50%), always remaining above.

In none of the sets, the significance of any variable stands out.

TCGA set: Tables 10 and 11.

### 2.7. Study of the Effects of Chemotherapy and Hormone Therapy

The first task that we carried out as part of this project was an analysis of survival and the performance utility of hormonal therapy and chemotherapy requested by the doctor who provided us with the data for the Hospital set.

For this reason, this task is carried out only with the original (and cleaned) variables of this set and the corresponding groupings of the paper with which the results are compared [10].

#### 2.7.1. Utility or Performance Assessment Measures

RR: relative risk of death of patients receiving treatment relative to those exposed to treatment not exposed to treatment.

RR: relative risk reduction. The percentage that the treatment reduces the risk of death. RRR = (1 − RR)∗100.

RRI: relative increase in risk.

RRI = ARI.

ARR: absolute risk reduction, percentage of people in whom death can be avoided by applying the treatment. ARR = (not exposed to treatment − exposed to treatment)∗100.

NNT: necessary number of patients to treat to reduce an event (recurrence). NNT = 1.

ARI: absolute increase in risk. ARI = experimental rate − control group rate.

NNH: number of patients that need to be treated for a patient to suffer an adverse event. NNH = 1.

#### 2.7.2. Chemotherapy Performance

As we can see in Table 7 and as observed in the paper, exposure to chemotherapy increases the death rate significantly, the more severe the patient is.  Table 12 shows that chemotherapy does not reduce the risk of death, but quite the contrary, for this reason, it does not make sense to calculate the necessary number of patients to expose to chemotherapy to reduce an event (NNT).

We see in Table 13 that in the Kaplan-Meier method, we reject the hypothesis that chemotherapy treatment does not cause effects on survival with a value = 3*e* − 04. With the Cox estimator, we see that the chemotherapy variable has an impact coefficient of 0 and 84, a risk index of 2.33 with a standard error of 0.24, and a *p* value of 0.0004.

#### 2.7.3. Hormone Therapy Performance

With the minimum positive number of patients to be treated to avoid a case of recurrence, we have aromatase inhibitors (AI) as the best treatment, followed by this combined with Tamoxifen.  Table 14. At the doctor's recommendation, we stopped working with the chemotherapy variable from the beginning.

### 2.8. Proposal of Hormonal Treatment Based on the Expiration

#### 2.8.1. Data Replication

Machine learning algorithms learn by understanding the relationship between the predictor variables and the variable to predict in order to create a pattern. Furthermore, whatever the size of the data, it is a small fraction of the global population, and in nature, there are always fluctuations that differ from a strict pattern. Our objective is to find the pattern of the entire population with a sample of size *N*, and the larger *N*, the smaller the differences with the overall population.

Our two sets of 827 and 648 records are very small and insufficient to represent the global population, so it is necessary to replicate them before they can be used to train a model.

#### 2.8.2. The Data Replication Algorithm Designed Consists of, for each Record

Its event and tracking time (in months) is stored. A start time and an interval are assigned according to the follow-up time: if it is greater than 10 months, the start time will be 10 months prior to that month; if not, it will be 0. The interval will be one day, each part of the difference between the end time and follow-time.

- From its defined start time to follow-up time and with interval 4 if it is the Hospital dataset or 3 if it is the TCGA dataset, the rest of the variables will be replicated with the unobserved event for each time
- If the event has taken place (event = 1), from follow-up time to the maximum time of that set and with the calculated interval, the rest of the variables are replicated

The main idea is that a patient with time *t* ∈ [0, *T*] had not suffered the event in time *t*_*i*_ ≤ *t*, and if he has suffered it at time *t*, he would also have suffered it for a time *t*_*i*_ ≥ *t*. In the records that replicate in backward time, they only do so up to a proportional time, and those that go to the end also do so with an interval proportional to their position. In addition, we have made the interval that replicates the data with event = 1 smaller to reduce the possibly problematic initial bias of the event variable. As we can see in the graphs contained in the annexed documents of the project and not exposed here because there are too many, the frequency distributions of all the variables are kept almost perfectly for both sets. The most important distribution to maintain is the distribution of events over time. In Table 15, we can see how by maintaining the distributions; we have managed to reduce the censored data by 17% and 12%.

#### 2.8.3. Using *mlr*: Choice of Predictor Type

Having the data ready to use a prediction model, we will do an exploration to find out which type of predictor is the most appropriate. We will explore the functioning of survival-type predictors (those used in a standard way in this type of study) and predictors of probability classification. The latter, for each level of the variable to be predicted (0 or 1), will calculate its probability and return the most probable as prediction.

For this exploration, we will use the *mlr* package for R [11]. This package (acronym for machine learning in r) provides an infrastructure that, using resampling methods, evaluates the indicated algorithms making an internal adjustment to find the best hyperparameters in each case.

To use this framework, we introduce the task and learner concepts. The tasks encapsulate the data and information about it necessary for the machine learning algorithm. We will create them with the functions makeSurvTask () indicating the tracking time variable and the event and makeClassifTask () indicating the variable event-to and the level that defines the survival. The learners contain the properties of the methods, we create them with the makeLearner () function, and we will indicate the algorithm and type of prediction in each case. We will also define the characteristics of the resampling strategy with the makeResampleDesc () function. In our case, we have chosen cross-validation with *k* = 5. Finally, with the function resample (learner, task, and resampling) indicating the parameters created previously, we will obtain the mean validation measures of the validation set in the iterations of the resampling algorithm. For both sets, we will test their available algorithms in each case.

#### 2.8.4. Survival Predictors

We evaluate it with the measure C-index 2.2.3. As we have seen in the explanation of this metric, a value less than 0.7 defines the model as very weak and inconsistent. None of the algorithms give good results, and the ones that are somewhat better have a high execution time. The TCGA set performs better on this type of predictor than the Hospital set. We can see the results in Table 16.

#### 2.8.5. Predictor Probability Classification

We evaluate them with measures ACC and MMCE 3.2.1. In these predictors, we also agree on the best performance over the TCGA set, although for both sets the results are notably better than those of the survival predictors, and they present more stable execution times between the different algorithms. We can see the results in Table 17. We highlight the good performance of the Bart machine algorithm (Bayesian additive regression trees) over the rest, so we will focus on exploring the algorithms derived from decision trees (random forest and gradient boosting).

#### 2.8.6. Using *h2o*

Exploratory analysis of classification models: once we know from the previous step that we are going to use predictors of the probabilistic classification type, we will use the *h2o* library in R [12]. This open platform offers parallel implementations of computational learning algorithms. We will use it to automate the training process of the algorithms (deep learning, random forest, gradient boosting machine, and extreme gradient boosting machine). In the previous section, we have seen the good performance of the algorithms derived from decision trees, but we will also check the behavior of the well-known deep learning algorithm.

As in the analysis in the previous section, we will also evaluate the mean measures of the validation set in a cross-validation *k* = 5. These measures will be calculated from the difference between the predictions. On returned (0 or 1) with the actual event value. Once we have validated a model, as this is a probabilistic type, we will be able to access the probability that the output is 0, that is, the probability of survival. Are probabilities for the different times will define a survival curve? Given that the unbalance in the levels in the variable to be predicted is remarkable, as we have seen in Table 15 and Figure 1, we will test the models with the balanced and unbalanced event variable for both sets.

#### 2.8.7. Hormone Therapy Decision Based on Predicted Survival

Using the Shiny extension for R, we will create an interface. In this interface, it is possible to enter the clinical data of the patient available in each set in the form of the finally chosen groupings, in addition to a fixed time. Making use of the models finally chosen and validated for each set, we will predict for the data entered the probability of survival (of which event has the value 0) for each time, returning a survival curve. In the case of the Hospital group, in which we have had the hormone therapy variable with the values IA, Tamoxifen, and Tamoxifen+IA for training, we will be able to see differentiated survival curves for each of the treatments, thus being able to know which is the one that maximizes survival in each particular case. The exact survival values for the fixed time entered will also be returned.

## 3. Results

Tables 18–21 show result details as follows.

Hospital set. Mean results of the validation set with classification predictors.

TCGA set.

### 3.1. Survival Curves

In the following figure, the survival curve of the unreplicated dataset is presented in the upper part. At the bottom left is the replicated set and to the right the predicted events from the replicated set and the predictor model chosen for each set.

## 4. Discussion

Our first objective was to analyze the usefulness and performance of hormone therapy and chemotherapy as treatments in our patients with adjuvant therapy and positive hormone receptors (Figure 2). We have seen that hormonal therapy (especially that containing aromatase inhibitors) is well accepted and can significantly improve survival. On the other hand (Figure 3), chemotherapy, far from being effective and reducing the risk of relapse into the disease, increases it in those patients who are exposed to this treatment. Furthermore, the risk of relapse has been greater the severity of the patient.

The second objective was to discover whether, for the numerical variables of our sets, the stratifications created by unsupervised machine learning that adapt to the data better explain the risk of death and recurrence than those used in a standard way. Walk in clinical practice. Having analyzed the best clustering option for each case, and analyzed these with the semiparametric Cox and nonparametric Kaplan-Meier statistical methods, we have obtained the expected results. In the case of the TCGA set with only two numerical variables, both have given their greatest significance in the stratifications defined by the *K-means* algorithm. In the case of the Hospital group, the most significant stratifications are divided between those used in the paper and those obtained by the clusters. For both sets, it is true that the standard stratifications in no case are the ones that best explain the risk. Once the sets with the chosen variables were defined, we wanted to find an accurate survival predictor using machine learning algorithms and check its improvement with respect to traditionally used statistical methods. We had estimated that we would obtain better results with computational learning methods than with statistical methods. We had also estimated that our data processing would improve with respect to the results normally obtained in these types of problems. In the exploratory analysis carried out with *mlr*, we have seen that, for the statistical methods, the maximum *C-index* reached is 0.58 in the Hospital set and 0.7 in the TCGA set; however, the computational learning approaches find their minimum value at a precision of 0.83 in the Hospital set and 0.82 in the TCGA set. Regarding the statistical predictors found in the literature, we can see in some examples that our results are not far from the real paradigm in cases of breast cancer obtained a maximum C-index of 0.629 in predicting the risk of recurrence. Also, with a statistical method, obtain a maximum AUC of 0.740, which obtain maximum AUCs of 0.791 and 0.714, respectively. Regarding the results with computational learning approximations in breast cancer, our validation results for the Hospital set find a maximum AUC of 0.974 (with a 0.003 standard error) with DL for the set Hospital and 0.962 (with a standard error of 0.005) with XGBoost for the TCGA set. Regarding the examples found in the literature of the last years with this approximation, we found a maximum AUC of 0.86 with ML-RO predictors, 0.930 with RF or 0.936 with DL and RF in a study using more than 200,000 cases and claimed to be the best outcome to date in 2005 [13].

Not only can we affirm that, indeed, computational learning approaches significantly exceed the precision that can be obtained with statistical approximations in risk prediction in breast cancer patients; if not that, in addition, our results obtained from replicated data with stratifications adjusted with machine learning seem to surpass those studies in which this step is not performed.

## 5. Conclusion

Within our own results, we can see how, in both sets, the precision results obtained from the same original set, having replicated and chosen the stratifications, clearly differ from those obtained in the est' version walk and without replicating. The precision in automatic learning algorithms increases between 20% and 30% thanks to the treatment carried out. In the Hospital set, the algorithm that works best is DL, probably due to having more data and being able to take advantage of its complexity (we check it in the set without replicating, where DL has the worst results among the algorithms analyzed). In the TCGA set, with less data and slightly lower results, the best performance is obtained with the XGBoost algorithm with little difference with respect to DL.

It is also noteworthy that the precision values per class are lower than the global ones due to the large difference in frequency in the levels of the variable to be predicted. Due to this difference, we have performed the same analysis balancing the data. In the Hospital group, we can see an improvement in the precision values, although their standard error ranges are generally the worst. In the TCGA set, the differences caused by the balancing of data are almost imperceptible. Regarding the computation, we have not found any impediment thanks to the stoppage offered by *h2o*. If we did not have it, it is likely that we would not have reached such precise results, or not with the same effort.

## Figures and Tables

**Figure 1:** Interface preview (^∗^CTS5 refers to the Hospital set).

**Figure 2:** TCGA joint survival curves for the entire population.

**Figure 3:** Hospital whole population survival curves.

**Table 1:** Variable numerical aggregations.

Variable	Standard grouping	Grouping paper	Applicable and clusterisable in dataset
Age	≤50, >50	Disaggregated	Hospital and TCGA
Nodal state (lymph nodes affected)	0, 1, 2-3, 4-9, +9	0, 1, 2-3, 4-9, +9	Hospital and TCGA
Tumor stage (tumor size in mm)	0, 0-20, 20-50, >50	<10, 10-20, 20-30, >30	Hospital
Ki67 concentration	≤14, >14	<10, 10-20, >20	Hospital
Lymph nodes removed	—	—	Hospital

**Table 2:** Summary datasets.

Dataset	Number of records	Number of predictive variables	Number of records censored	Maximum event time	Event meaning
Hospital	874	12	738 (89%)	26 years	Recurrence
TCGA	648	8	584 (90%)	13 years	Death

**Table 3:** Hospital variable quality analysis from *p* value and 95% CI.

Variable	*p* value Kaplan-Meier	Kaplan-Meier 95% CI	*p* value Cox PH
Disaggregated age	<0.0001	0.576-0.999	0.4
Standard age	0.86	0.854-0.933	0.9
Age K-means *k* = 4	0.37	0.831-0.943	0.4
Disaggregated affected lymph nodes	<0.0001	0.725-0.96	0.005
Standard and paper affected nodes	<0.0001	0.771-0.942	<0.0001
Lymph nodes affected K-means *k* = 2	0.0063	0.843-0.929	0.01
Hierarchical lymph nodes *k* = 3	<0.0001	0.811-0.927	<0.0001
Lymph nodes removed disaggregated	0.0005	0.642-0.987	0.005
Hierarchical nodes *k* = 4	0.074	0.825-0.937	0.06
Disaggregated tumor size	<0.0001	0.648-0.982	0.1
Standard tumor size	0.07	0.838-0.935	0.08
Tumor paper size	0.027	0.823-0.939	0.03
Hierarchical tumor size *k* = 20	0.2	0.852-0.932	0.2
Tumor size K-means *k* = 3	0.07	0.837-0.936	0.07
Ki67 disaggregated	<0.0001	0.642-0.988	0.5
Ki67 standard	0.46	0.854-0.933	0.5
Ki67 paper	0.44	0.841-0.943	0.5
Ki67 hierarchical *k* = 7	0.68	—	0.7
Hormone receptor	0.79	0.855-0.931	0.8
Menopausal state	0.71	0.855-0.9331	0.7
Degree	0.43	0.842-0.935	0.4
Cancer subtype	0.29	0.854-0.933	0.3
Risk	0.0001	0.825-0.919	<0.0001
Hormone therapy	0.011	0.836-0.943	0.02

**Table 4:** Hospital joint Cox proportional hazards test.

Set	Rho global estimator	Global Chi estimator	Global *p* value
Standard	0.037	0.54	1
Paper	NA	0.38	1
Combined	NA	0.5	1

**Table 5:** Tests global significance variables Cox PH model sets Hospital.

Set	Global likelihood test	Wald global test	Global LogRank test
Standard	<2^−16^	0.9	<2^−16^
Paper	<2^−16^	0.9	<2^−16^
Combined	<2^−16^	1	<2^−16^

**Table 6:** Quality analysis of TCGA variables from *p* value and 95% CI.

Variable	*p* value Kaplan-Meier	95% CI Kaplan-Meier	*p* value Cox PH
Disaggregated age	<0.0001	0.489-1	<0.0001
Standard age	0.0014	0.82-0.93	0.0004
Age K-means *k* = 3	<0.0001	0.789-0.95	<0.0001
Age K-means *k* = 4	<0.0001	0.777-0.955	<0.0001
Disaggregated affected lymph nodes	0.54	0.612-0.998	0.4
Standard and paper affected nodes	0.006	0.788-0.965	0.02
Lymph nodes affected K-means k = 3 + neg	0.001	0.785-0.967	0.004
Lymph nodes affected K-means *k* = 4	0.61	0.796-0.962	0.6
Menopausal state	<0.0001	0.816-0.924	<0.0001
Tumor stage	0.00029	0.809-0.942	0.001
Tumor stage	<0.0001	0.788-0.96	0.01
Hormone receptor	0.44	0.803-0.949	0.5
Cancer subtype	0.18	0.798-0.958	0.2

**Table 7:** Impact index, standard error, risk index, *p* value, and 95% confidence intervals using the Cox model in conjunction with TCGA.

Variable	Impact coefficient	Hazard ratio	Standard error	*p* value	95% CI (RH)
Premenopausal	1.35	3.8	3.168	0.66	7*e* − 03 (1.930e+03)
Luminal A	-1.05	0.34	4709	0.99	0 (Inf)
Luminal B	1.64	0.19	4709	0.99	0 (Inf)
Stage II tumor	-0.97	0.37	2.89	0.73	1.294*e* − 03 (1.105*e* + 02)
Stage III tumor	-0.16	0.85	2.54	0.94	5.852*e* − 03 (1.238*e* + 02)
Stage IV tumor	-7.27	6.90*E* − 04	2.00*E* + 04	0.99	0(Inf)
Hormone receptor EP	-1.18	0.3	2.36	0.62	3.011*e* − 03 (3.132*e* + 01)
Hormone receptor other	-2.94	0.05	4709	0.99	0(Inf)
Hormone TN receptor	-2.67	0.07	4709	0.99	0 (Inf)
Age (54.70]	-0.48	0.61	3.75	0.89	3.871*e* − 04 (9.709*e* + 02)
Age (70,100]	0.08	1.08	3.29	0.97	1.693*e* − 03 (7.004*e* + 02)
Nodal status (0.8]	1.43	4.19	2.3	0.53	4.58*e* + 02 (3.83*e* + 02)
Nodal status (19.44]	1.3	3.68	2.38	0.58	3.446*e* − 026 (3.931*e* + 02)
Nodal status (8.19]	0.35	1.42	2.2	0.87	1.798*e* − 02 (1.132*e* + 02)

**Table 8:** Hospital correlation hypothesis tests.

Observed correlation	Correlation index	*p* value test	Hypothesis
Nodal state and risk	0.82	0.06	*H*_0_
Age and menopausal status	0.75	0.3	*H*_0_
Tumor size and risk	0.51	0.004	*H*_1_

**Table 9:** Tests of hypothesis TCGA correlations.

Observed correlation	Correlation index	*p* value test	Hypothesis
Cancer subtype and hormone receptor	0.43	0.6	*H*_0_
Menopause and age	-0.67	0.002	*H*_1_

**Table 10:** Kaplan-Meier survival adjustment of the Hospital set and TCGA.

	*n*	Events	Median	SD average	Median	95% CI
Hospital	826	88	21.82	0.42	NA	NA
TCGA	648	64	10.03	0.41	10.23	9.51

**Table 11:** Impact index, standard error, risk index, *p* value, and 95% confidence intervals using the Cox model as a whole Hospital.

Variable	Impact coefficient	Hazard ratio	Standard error	*p* value	95% CI (RH)
Postmenopausal	-3.54	0.28	6.08	0.56	1.9*e* − 07 (4370)
Luminal B	-0.76	0.46	3.14	0.81	9.8*e* + 04 (222)
Intermediate risk	-0.59	0.55	0.89	0.88	1.6*e* + 04 (222)
High risk	-2.15	1.97	6.52	0.74	3.2*e* − 07 (1850)
Tamoxifen	-2.35	0.12	3.39	0.49	1.2*e* − 04 (4.15*e* + 04)
Tamoxifen-IA	-1.73	0.18	4.01	0.66	6.8*e* − 05 (73.3)
Tumor size (10.20]	-2.09	0.12	3.81	0.58	7.05*e* − 5 (218)
Tumor size (20,30]	0.22	1.25	5.01	0.96	7.05*e* − 05 (2.29*e* + 04)
Tumor size (30,100]	-2.18	0.11	4.38	0.62	6.81*e* − 05 (602)
Ki67 borderline	2.05	7.78	4.92	0.68	4.98*e* − 04 (1.21*e* + 05)
Ki67 high	2.11	8.23	4.04	0.6	0.003 2 (27e + 04)
Hormone receptor EP + RP	1.48	4.39	4	0.71	1730 1.1(1e + 04)
Age (44.56]	2.16	8.66	5.63	0.7	1.37*e* − 04 (5.45*e* + 05)
Age (56.69]	3.48	32.35	6.41	0.58	1.13*e* − 04 (9.23*e* + 06)
Age (69,100]	3.76	43.11	8.4	0.65	3.03*e* − 06 (6.13*e* + 08)
Nodal status (0.10]	0.88	2.41	4.49	0.84	3.66*e* − 04 (1.58*e* + 04)
Nodal status (10.25]	1.35	3.87	6.5	0.83	1.13*e* − 05 (1.31*e* + 06)
gg extracted (1.11]	1.05	2.84	4.42	0.81	4.86*e* − 04 (1.66*e* + 04)
gg extracted (11.17]	1.27	3.57	4.57	0.78	4.60e − 04 (2.77e + 04)
gg extracted (17.32]	8.17	1.08	5.61	0.98	1.82*e* − 05 (6.46*e* + 04)

**Table 12:** Death rate by risk group according to exposure to joint chemotherapy Hospital.

Risk group	Exposed chemotherapy	Unexposed chemotherapy
Global	14%	5.90%
Low	6%	5.40%
Intermediate	7.70%	5.50%
High	19%	7.40%

**Table 13:** Assessment of the utility of exposure to chemotherapy.

Risk group	RRR	NNT
Low	-10.90%	-167
Intermediate	-36.50%	-49
High	-157.30%	-9

**Table 14:** Acceptance of hormone therapy treatments.

Hormone therapy treatment	Control group rate	Experimental group rate	NNT	NNH
AI	0.106	0.105	19	-19
Tamoxifen	0.101	0.121	-53	53
AI+Tamoxifen	0.108	0.045	30	-30

**Table 15:** Joint states before and after replication.

Set	Initial size	Size after replication	Initially censored	Censored after replication
Hospital	827	3422	738 (89%)	2454 (72%)
TCGA	648	3137	584 (90%)	2433 (78%)

**Table 16:** Survival classifier results using *mlr* Hospital and TCGA.

	Algorithm	C-index	Execution time
Hospital	*CV CoxBoost*	0.58	8.6 min
	*CoxBoost*	0.58	1.8 min
	*CoxPH*	0.57	1 sec
	*CV Glmnet*	0.5	6 secs
TCGA	*CV CoxBoost*	0.7	7.2 min
	*CoxBoost*	0.69	26 secs
	*CoxPH*	0.68	0.2 secs
	*CV Glmnet*	0.62	4 secs

**Table 17:** Classifying results classification using *mlr* Hospital and TCGA.

	Algorithm	ACC	MMCE	Execution time
Hospital	*Bart machine*	0.88	0.12	1.3 mins
	*AdaBoost machine*	0.83	0.17	0.32 secs
	*Binomial*	0.85	0.15	0.2 secs
CGTA	*Bart machine*	0.99	0.1	62 secs
	*AdaBoost machine*	0.89	0.11	0.3 secs
	*Binomial*	0.82	0.14	0.7 secs

**Table 18:** Results with standard deviation of predictor classification using *h2o* in Hospital.

Algorithm	AUC	ACC	Average ACC per class	MSE	Average MSE per class
*Hospital with standard variables and without replication*					
DL	0.628 ± 0.044	0.543 ± 0.095	0.658 ± 0.032	0.146 ± 0.025	0.342 ± 0.032
XGBoost	0.692 ± 0.040	0.789 ± 0.112	0.650 ± 0.022	0.094 ± 0.013	0.349 ± 0.022
GBM	0.658 ± 0.043	0.767 ± 0.054	0.661 ± 0.056	0.106 ± 0.016	0.339 ± 0.056
RF	0.654 ± 0.039	0.763 ± 0.104	0.649 ± 0.027	0.097 ± 0.015	0.351 ± 0.027
*Replicated and unbalanced Hospital*					
DL	0.974 ± 0.002	0.926 ± 0.006	0.911 ± 0.005	0.059 ± 0.002	0.089 ± 0.005
XGBoost	0.964 ± 0.003	0.915 ± 0.006	0.888 ± 0.005	0.065 ± 0.002	0.112 ± 0.005
GBM	0.963 ± 0.003	0.915 ± 0.005	0.882 ± 0.005	0.066 ± 0.002	0.118 ± 0.005
RF	0.961 ± 0.003	0.916 ± 0.005	0.881 ± 0.005	0.069 ± 0.002	0.119 ± 0.005
*Replicated and balanced Hospital*					
DL	0.974 ± 0.003	0.931 ± 0.005	0.917 ± 0.005	0.010 ± 0.003	0.082 ± 0.010
XGBoost	0.966 ± 0.005	0.925 ± 0.005	0.898 ± 0.010	0.061 ± 0.005	0.102 ± 0.010
GBM	0.965 ± 0.006	0.921 ± 0.011	0.889 ± 0.005	0.010 ± 0.006	0.111 ± 0.010
RF	0.965 ± 0.004	0.922 ± 0.007	0.902 ± 0.008	0.067 ± 0.006	0.098 ± 0.008

**Table 19:** Higher precision model for Hospital set: deep learning with balanced data, hyperparameters. Learning rate = 0.005, 2611 epochs.

Cap	Activation function	Units	*Dropout index*
Entry	—	—	15%
Hidden 1	*Rectifier dropout*	500	50%
Departure	*Softmax*	2	—

**Table 20:** Results with standard deviation of predictor classification using h2o in TCGA.

Algorithm	AUC	ACC	Average ACC per class	MSE	Average MSE per class
*Standard variables and without replication*					
DL	0.591 ± 0.019	0.706 ± 0.076	0.639 ± 0.024	0.147 ± 0.032	0.361 ± 0.024
XGBoost	0.631 ± 0.029	0.695 ± 0.101	0.634 ± 0.038	0.091 ± 0.012	0.366 ± 0.037
GBM	0.647 ± 0.046	0.826 ± 0.038	0.639 ± 0.035	0.109 ± 0.017	0.361 ± 0.035
RF	0.642 ± 0.046	0.806 ± 0.081	0.629 ± 0.036	0.090 ± 0.014	0.371 ± 0.036
*Replicated and unbalanced TCGA*					
DL	0.961 ± 0.009	0.925 ± 0.004	0.883 ± 0.010	0.064 ± 0.005	0.117 ± 0.010
XGBoost	0.962 ± 0.005	0.929 ± 0.004	0.897 ± 0.009	0.055 ± 0.003	0.102 ± 0.009
GBM	0.961 ± 0.005	0.929 ± 0.006	0.892 ± 0.012	0.056 ± 0.002	0.108 ± 0.012
RF	0.959 ± 0.005	0.926 ± 0.004	0.882 ± 0.003	0.061 ± 0.002	0.118 ± 0.003
GLM	0.933 ± 0.007	0.890 ± 0.018	0.859 ± 0.005	0.109 ± 0.006	0.143 ± 0.013
*Replicated and balanced TCGA*					
DL	0.961 ± 0.009	0.925 ± 0.004	0.882 ± 0.010	0.064 ± 0.005	0.117 ± 0.010
XGBoost	0.961 ± 0.005	0.929 ± 0.004	0.897 ± 0.009	0.056 ± 0.003	0.108 ± 0.012
GBM	0.962 ± 0.005	0.929 ± 0.006	0.892 ± 0.012	0.056 ± 0.002	0.108 ± 0.012
RF	0.959 ± 0.005	0.926 ± 0.004	0.882 ± 0.003	0.061 ± 0.002	0.118 ± 0.003
GLM	0.933 ± 0.007	0.890 ± 0.010	0.859 ± 0.005	0.019 ± 0.006	0.143 ± 0.013

**Table 21:** Higher precision model for TCGA set: extreme gradient boosting with unbalanced data, hyperparameters. 160 epochs.

Number of trees	153
Max deep	15
*Learning rate*	5

## Data Availability

The data used to support the findings of this study are included within the article.
